# Peptides Released from Foremilk and Hindmilk Proteins by Breast Milk Proteases Are Highly Similar

**DOI:** 10.3389/fnut.2017.00054

**Published:** 2017-11-02

**Authors:** Søren D. Nielsen, Robert L. Beverly, David C. Dallas

**Affiliations:** ^1^Nutrition Program, School of Biological and Population Health Sciences, College of Public Health and Human Sciences, Oregon State University, Corvallis, OR, United States

**Keywords:** peptides, human, mother’s milk, casein, whey, bioactive, protease

## Abstract

Human milk contains active proteases that initiate hydrolysis of milk proteins within the mammary gland. Milk expressed at the beginning of feeding is known as foremilk and that at the end of feeding is known as hindmilk. As hindmilk contains higher fat, vitamins A and E, and higher calories than foremilk, feeding only hindmilk initially and reserving foremilk for later are practiced in some neonatal intensive care units. This study investigated the difference in peptide profiles, predicted milk protease activities, and bioactive peptides between foremilk and hindmilk. Bioactive peptides are short fragments of proteins that influence biological processes. Four mothers pumped 10 mL of their foremilk and 10 mL of their hindmilk into iced containers prepared with antiproteases and the samples were immediately frozen. The peptide profile of each sample was analyzed by liquid chromatography nano-electrospray ionization Orbitrap Fusion tandem mass spectrometry. Peptide abundance (sum of ion intensities) and count (number of unique peptide sequences) in each milk sample were determined from this analysis. The specific enzymes that participated in peptide release were predicted based on the amino acids positioned at each cleavage site. Peptide bioactivity was predicted based on homology to a known functional peptide database and two bioactivity prediction algorithms. Hindmilk contained a higher count of peptides than foremilk. The higher number of unique peptide sequences in hindmilk was related to hydrolysis of β-casein, osteopontin, α_s1_-casein and mucin-1 via plasmin and elastase cleavage, and possible aminopeptidase and carboxypeptidase activities. Though hindmilk contained a greater number of peptides than foremilk, the overall peptide abundance did not differ and most of the total peptide abundance derived from peptide sequences that were present in both milk types. The presence of higher numbers of predicted bioactive peptides in the hindmilk could indicate that the practice of providing hindmilk rather than foremilk to premature infants could positively impact health outcomes; however, as there are few differences in overall peptide abundance, the overall effect is likely limited.

## Introduction

Human milk has evolved to match the newborn infant’s nutritional needs and is highly important for the growth and development of the neonate. Besides providing the infant with nutrients, human milk contains many bioactive components that are preformed prior to expression, such as immunoglobulins, hormones, and growth factors, that contribute to the infant’s development. In addition to proteins that are bioactive intact, milk proteins contain encrypted sequences released upon proteolysis that exert an array of functions, often different from that of the parent protein.

Breastfeeding has been associated with a number of health benefits for the human infant, such as reduced risk of non-specific gastroenteritis, severe lower respiratory tract infections, type 1 and 2 diabetes, and necrotizing enterocolitis (1). Though the mechanisms for these associations are not entirely clear, they are likely due to the coordinated effects of the bioactive molecules in milk. Milk protein-derived peptides have an array of identified functions that may benefit the infant, including antimicrobial, immunomodulatory, angiotensin-converting enzyme (ACE)- and dipeptidyl peptidase IV inhibitory, and opioid activity (2–4).

Our recently constructed online database of all known bioactive milk peptides (5) contains hundreds of peptides that have been experimentally confirmed as bioactive. Many of these peptides were identified from human milk samples after *in vitro* digestion with gastric enzymes (6–8) or selected for testing by applying predictive models to the entire milk protein sequences (9, 10).

Previous literature demonstrated that human and bovine milks contain an array of proteases and protease inhibitors [reviewed in Ref. (11)]. Our recent work confirmed that native proteases exist in milk, including (from highest to lowest concentration) carboxypeptidase B2, plasmin, kallikrein, elastase, thrombin, cathepsin D, and cytosol aminopeptidase. Besides cathepsin D, which is inactive at milk pH, all of these milk proteases are in active forms within milk (12). The presence of numerous proteases in milk is proposed to lead to hydrolysis of the milk proteins (11–13). In previous studies, peptides derived from the natural proteolysis of milk proteins have been identified (7, 14–17). This intra-mammary gland proteolytic activity can occur in the time between milk expressions for feeding the neonate, in which milk is secreted from mammary epithelial cells and stored in alveoli and lactiferous ducts until expression (18). The native proteolytic activity of milk may release peptides that are relevant to the developing infant or the mammary gland itself.

Previous studies have demonstrated differences in the composition of milk expressed at the beginning of feeding (foremilk) and end of feeding (hindmilk). Foremilk has been defined as the first 2–3 min after flow initiation (“letdown”) and hindmilk is defined as the remainder of milk obtained until complete breast emptying (19, 20). Hindmilk has a higher fat concentration, energy density, and concentration of vitamins A and E (19, 21, 22). These previous studies were performed with sample sizes of between 15 and 24 mothers. Though there is little significant difference in protein content between foremilk and hindmilk (23), hindmilk resides longer within the mammary gland in the presence of the native milk proteases than foremilk, thus potentially affecting the peptide composition of the milk. Such changes could alter the availability of bioactive peptides for the infant.

Based on previous results showing differences in the nutritional composition between foremilk and hindmilk, and due to the activity of native milk proteases, we hypothesized that the count and abundance of milk peptides between foremilk and hindmilk would be different as well. Foremilk and hindmilk from four term mothers were analyzed via mass spectrometry-based peptidomics and examined for differences in peptides, predicted protease activity, and predicted bioactive peptides.

## Materials and Methods

### Participants and Samples

The study was approved by the Institutional Review Board at Oregon State University, and informed consent was obtained from all mothers. Human foremilk and hindmilk samples were collected from four mothers (2–4 months of lactation). All mothers gave birth to term infants. Mothers with any signs of clinical mastitis and current antibiotic usage were excluded from the study. Before pumping, mothers thoroughly washed their hands and cleansed their nipples with a moist single-use paper towel. Breasts were pumped using a hospital-grade Medela Symphony electrical pump (Salem, OR, USA). All parts that contacted the mother or her milk were single use. Mothers were instructed to pump the first 10 mL of milk (foremilk) into an 80-mL breastmilk collection container (6109S-100; Medela) premarked at the 10-mL line. The container was prepared with protease inhibitor solution and held on ice [1 tablet of a protease inhibitor cocktail (cOmplete™ mini protease inhibitor cocktail tablets, 11836153001; Roche, Basel, Switzerland) added to 1 mL of MilliQ water, according to the manufacturer’s instructions]. The exact components of the antiprotease mixture are not disclosed; however, it inhibits a wide array of serine, cysteine, and metalloproteases as well as calpains. When the level of milk reached 10 mL, the mother immediately stopped pumping and passed the milk bottle to the researchers. The milk was immediately mixed well by gentle rocking, and divided into five 2-mL aliquots in 2-mL Eppendorf tubes and placed on dry ice within 1 min after expression. The mother kept pumping the milk into a second container until the flow rate dropped and the mother felt her breast was near empty [in all cases, later than 3 min after flow initiation, the standard definition for hindmilk (19)]. The mother then pumped 10 mL of hindmilk into a third container, which was handled as described for foremilk. After removing aliquots, the samples were immediately transported on dry ice to storage in a −80°C freezer within 30 min of expression. Milks were stored at −80°C for a maximum of three weeks prior to peptidomic analyses.

### Sample Preparation

Aliquots of each milk sample (four foremilk and four hindmilk samples) were thawed on ice for approximately 30 min before removing the milk fat by centrifugation (3,000 × *g* for 10 min at 4°C). The infranates (400 µL) were collected by pipette. Milk proteins were precipitated from the skimmed milk by adding 400 µL of 24% trichloroacetic acid (240 g/L) followed by agitation of a vortex mixer for 10 s. Samples were centrifuged at 4,000 × *g* for 10 min at 4°C, and 600 µL of the supernatant containing the peptides were collected.

To remove trichloroacetic acid, salts, oligosaccharides and lactose from the peptide solution, the peptides were extracted via C18 reverse-phase preparative chromatography in 96-well plates (Glygen, Columbia, MD, USA). In general, unless otherwise noted, the volume of solution used in the different steps was 200 µL and the centrifuge parameters were 2,000 × *g* for 1 min at 4°C. Each step was repeated three times. To activate the C18 reverse-phase columns, 99% acetonitrile (ACN), 0.1% trifluoroacetic acid (TFA) solution was added. Columns were equilibrated with 1% ACN, 0.1% TFA before each sample was added to a separate well and centrifuged. This step was repeated two more times to load the total sample volume (600 µL) onto the column. The columns were washed with 1% ACN, 0.1% TFA to remove trichloroacetic acid, salts, lactose and oligosaccharides. The peptides were eluted with 80% ACN, 0.1% TFA. The peptide solutions were lyophilized using a freeze dry system (Labconco FreeZone 4.5 L, Kansas City, MO, USA). After freeze drying the samples, they were rehydrated in 40 µL of 0.1% FA in water.

### Protein Determination

The bicinchoninic acid assay for protein (ThermoFisher Scientific, Waltham, MA, USA)—conducted as described by the manufacturer with bovine serum albumin as reference protein—was used for determination of the protein/peptide concentration (24).

### Liquid Chromatography Nano-Electrospray Ionization Mass Spectrometry Peptide Profiling

Liquid chromatography separation was performed on a Waters Nano Acquity UHPLC (Waters Corporation, Milford, MA, USA) with a nanospray source. Peptides were loaded (1 µL) onto a 180 µm × 20 mm, 5-µm bead 2 G nanoAcquity UPLC trap column (reverse-phase) for enrichment and online desalting and then onto a 100 µm × 100 mm, 1.7-µm bead Acquity UPLC Peptide BEH C18 column (Waters) connected to a Orbitrap Fusion Lumos (Thermo Scientific). To reduce the effects of analysis variation, the samples were loaded alternating between the two milk types. Peptides were eluted using a gradient of 0.1% FA in water (A) and 99.9% ACN, 0.1% FA (B) with a flow rate of 500 nL/min. The 120-min gradient consisted of 3−10% solvent B over 3 min, 10−30% solvent B over 99 min, 30−90% solvent B over 3 min, 90% solvent B for 4 min, 90−3% solvent B over 1 min then finally held at 3% solvent B for 10 min. Each sample analysis was followed by a 30-min column wash.

Spectra were collected in positive ionization mode with an electrospray voltage of 2,400 V. The mass spectrometer was set to scan masses between 400 and 1,500 *m*/*z* at a resolution of 120 K. The automatic gain control target was set to 4.0 × 10^5^, with a maximum injection time of 50 ms. The fragmentation mode was set to collision-induced dissociation and the collision energy was 35%. The mass spectrometer cycle time was 3 s, with data-dependent analysis and automated precursor peak selection. Precursors were excluded (10 ppm mass error) after one fragmentation and held for 1 min. Precursor ions were selected for fragmentation based on the following criteria: most intense peaks, ion intensity threshold 5.0 × 10^3^ and charge state 2–7. Fragments were detected with ion trap automatic scan range.

Spectra were analyzed by database searching in Thermo Proteome Discoverer (v2.1.0.81). The data were searched against an in-house human milk protein sequence database. Phosphorylation of serine and threonine and oxidation of methionine was allowed as potential modifications. Peptides identified with high confidence (*P* < 0.01) were accepted. Each peptide sequence with multiple modifications was grouped into a single entry for counts. Counts measured the number of unique peptide sequences identified in a sample. Abundance measured the area under the curve of the eluted peak (ion intensity). As the abundance measurement is based on relative ion intensity, it is only an approximation of the amount of peptides in the samples.

Peptides were mapped to their parent protein sequence of β-casein, osteopontin, and α_s1_-casein using an in-house tool (PepEx) (15), which can be accessed at http://mbpdb.nws.oregonstate.edu/pepex/. PepEx gives a visualization of the position of peptides identified by totaling the abundance or count of each amino acid from the peptidomic data.

### Bioactive Peptide Identification and Prediction

The identified peptides in human milk samples were investigated for literature-identified bioactive peptides using our recently created Milk Bioactive Peptide Database (MBPDB) (5), which is a comprehensive database of all milk protein-derived bioactive peptides reported in literature and can be accessed at http://mbpdb.nws.oregonstate.edu/. The search performed was conducted as a sequence search, which searches for bioactive peptides matching the input peptide sequence. To predict the bioactive potential of each identified peptide, we used two online prediction tools—CAMPR3 (antimicrobial prediction) (25) and Peptide Ranker (general bioactivity prediction) (26). The CAMPR3 prediction was conducted by inputting the list of identified peptide sequences and searching for antimicrobial potential with four algorithms (SVM, random forest, artificial neural network, and discriminant analysis). For general bioactivity (Peptide Ranker), peptide sequences were input with no further options available and results were scores from 0 to 1 for each peptide with 1 being most likely to be bioactive.

### Enzyme Prediction

To investigate which proteases were involved in cleaving human milk proteins into peptides, three approaches were used. In Proteome Discoverer, peptides were identified with annotated sequences. With this information, Excel was used to determine the count and abundance of which amino acids were present in the P1 and P1′ positions of the N- and C-termini of each peptide identified. The cleavage specificity of known milk proteases were mapped to these amino acids for visual interpretation in the figures [based on the most abundant amino acids listed at P1 and P1′ on Merops (27)] and included elastase (MEROPS ID: S01.131), kallikrein 6 (KLK 6) (MEROPS ID: S01.236), kallikrein 11 (KLK 11) (MEROPS ID: S01.257), plasmin (MEROPS ID: S01.233), and thrombin (MEROPS ID: S01.217). To determine which peptides were possibly released by exopeptidase activity, the number of peptides that differed from a related sequence by one amino acid at either the N- or C-termini was counted.

To predict which enzymes were active in milk using more complex cleavage specificity by accounting for amino acids from P4 to P2′ and P4 to P4′, the two online predictors EnzymePredictor and Proteasix, respectively, were used.

EnzymePredictor^1^ required input of the peptide amino acid sequences and their associated protein ID as found at uniprot.org (28). This information is used to identify the amino acids located at the P4, P3, P2, P1, P1′, and P2′ positions of both the N- and C-terminal cleavage sites of each peptide. Based on this information and the cleavage specificity patterns of the selected proteases, EnzymePredictor predicts which enzyme could yield each peptide. For each protease identified, EnzymePredictor provides the count of N-terminal-, C-terminal- and total cleavages assigned to each enzyme, the number of times an enzyme could have cleaved within all the protein sequences in the library of proteins observed and the odds ratio (comparing the number of predicted cleavages based on sequence alone with the actual peptide cleavages assigned to each protease).

Proteasix^2^ predicted which enzymes were involved in the peptide cleavage sites using amino acid cleavage patterns from Merops (27). Proteasix required the input protein ID and start and stop amino acid number of the peptide within the protein. The enzymes searched against were plasmin (PLG), neutrophil elastase (ELANE), thrombin (F2), KLK 6, and KLK 11 based on the amino acids positioned from P4 to P4′ at the cleavage site. Predicted and observed cleavages were combined in the result output.

### Statistical Analysis

Analyses were carried out using the statistical program RStudio version 1.0.136. A linear mixed model with Tukey’s HSD *post hoc* test was used to adjust for multiple comparisons between foremilk and hindmilk. Significant difference was defined as *P* < 0.05. Results are presented as least square mean ± SE. For individual comparison of the peptide abundance in foremilk compared to hindmilk, a two-tailed pairwise *t*-test was conducted using the *t*-test function in Excel.

## Results

### Peptide Profile

Protein concentration in breast milk was determined by the bicinchoninic acid assay and was not significantly different between the foremilk (10.2 ± 0.4 mg/mL) and hindmilk (9.5 ± 0.4 mg/mL). The coefficient of variation for total protein concentration was 8.6%. On average, 474 ± 14 peptides were identified in the foremilk and 591 ± 14 identified in the hindmilk (Figure 1A). Significantly more peptides were identified in the hindmilk than the foremilk (*P* = 0.0106). A total of 370.3 ± 11.7 peptides were found in both the foremilk and hindmilk of each mother and comprised 98.3 ± 1.1% of the foremilk peptide abundance and 96.7 ± 1.1% of the hindmilk peptide abundance. Of these peptides, 135 peptides deriving from 10 different proteins were identified in both fore and hindmilk of all four mothers (Tables 1–3). These accounted for 91.3 ± 3.5 and 86.8 ± 3.5% of the total abundance of peptides in foremilk and hindmilk, respectively. The abundance of all peptides in each sample were not significantly different between foremilk and hindmilk (5.9 × 10^11^ ± 7.1 × 10^10^ and 7.1 × 10^11^ ± 7.1 × 10^10^, respectively; Figure 1B). However, of all the peptides identified, 36 were found to be significantly more abundant in hindmilk than foremilk (*P* < 0.05; Table 4). No peptides were significantly more abundant in foremilk than hindmilk.

**Figure 1:** Total count **(A)** and abundance **(B)** of peptides in foremilk and hindmilk. Results are shown as least square mean ± SE, *n* = 4. Asterisks (*) indicate significant differences between foremilk and hindmilk (*P* < 0.05).

**Table 1:** Peptides derived from α_s1_-casein identified in both foremilk and hindmilk samples from all four mothers.

Sequence	Start	Stop
RPKLPLRYPE	16	25
RPKLPLRYPERLQNPSESSEPIPLESREEYMNGMN	16	50
RPKLPLRYPERLQNPSESSEPIPLESREEYMNGMNR	16	51
YPERLQNPSESSEPIPLESREEYMNGMN	23	50
RLQNPSESSEPIPLESREE	26	44
RLQNPSESSEPIPLESREEY	26	45
RLQNPSESSEPIPLESREEYMNGM	26	49
RLQNPSESSEPIPLESREEYMNGMN	26	50
RLQNPSESSEPIPLESREEYMNGMNR	26	51
LQNPSESSEPIPLESREEYMNGMN	27	50
NPSESSEPIPLESRE	29	43
NPSESSEPIPLESREEYMNGMN	29	50
EPIPLESREEYMNGMNR	35	51
QRNILREKQTDEIKDTR	52	68
RNILREKQTDEIKDTR	53	68
NILREKQTDEIKDT	54	67
NILREKQTDEIKDTR	54	68

*“Start” and “stop” indicate the amino acid numbers for the beginning and end of the peptide within the protein sequence (counting the signal sequence)*.

**Table 2:** Peptides derived from β-casein identified in both foremilk and hindmilk samples from all four mothers.

Sequence	Start	Stop
RETIESLSSSEESITEY	16	32
RETIESLSSSEESITEYK	16	33
RETIESLSSSEESITEYKQ	16	34
RETIESLSSSEESITEYKQK	16	35
RETIESLSSSEESITEYKQKVE	16	37
RETIESLSSSEESITEYKQKVEK	16	38
RETIESLSSSEESITEYKQKVEKVK	16	40
RETIESLSSSEESITEYKQKVEKVKHEDQQQGEDEHQD	16	53
RETIESLSSSEESITEYKQKVEKVKHEDQQQGEDEHQDK	16	54
RETIESLSSSEESITEYKQKVEKVKHEDQQQGEDEHQDKIYP	16	57
ETIESLSSSEESITE	17	31
ETIESLSSSEESITEYK	17	33
ETIESLSSSEESITEYKQ	17	34
ETIESLSSSEESITEYKQK	17	35
ETIESLSSSEESITEYKQKVEK	17	38
ETIESLSSSEESITEYKQKVEKVK	17	40
TIESLSSSEESITEYK	18	33
TIESLSSSEESITEYKQKVEK	18	38
IESLSSSEESITEYK	19	33
IESLSSSEESITEYKQKVEK	19	38
ESLSSSEESITE	20	31
ESLSSSEESITEYK	20	33
SLSSSEESITE	21	31
SLSSSEESITEYK	21	33
SLSSSEESITEYKQKVEK	21	38
LSSSEESITEYK	22	33
SSSEESITEYK	23	33
SSSEESITEYKQKVEK	23	38
SSEESITEYK	24	33
SSEESITEYKQKVEK	24	38
SEESITEYK	25	33
EESITEYK	26	33
QKVEKVKHEDQQQGEDEHQDKIYP	34	57
KVEKVKHEDQQQGEDEHQDKIYP	35	57
KVEKVKHEDQQQGEDEHQDKIYPS	35	58
VEKVKHEDQQQGEDEHQDKIYPS	36	58
VKHEDQQQGEDEHQDKIYP	39	57
VKHEDQQQGEDEHQDKIYPS	39	58
EDQQQGEDEHQDKIYPS	42	58
DQQQGEDEHQDKIYPS	43	58
LPVPQPEIMEVPKAKDT	91	107
AKDTVYTKGRVMPVLK	104	119
KDTVYTKGRVMPVLK	105	119
GRVMPVLKSPTIPFFDPQIPK	112	132
MPVLKSPTIPFFDPQIP	115	131
VLPIPQQVVPYPQ	176	188
LLNPTHQIYPVTQPLAPVHNPISV	203	226
NPTHQIYPVTQPLAPVHNPIS	205	225
NPTHQIYPVTQPLAPVHNPISV	205	226
YPVTQPLAPVHNPISV	211	226

*“Start” and “stop” indicate the amino acid numbers for the beginning and end of the peptide within the protein sequence (counting the signal sequence)*.

**Table 3:** Peptides derived from osteopontin identified in both foremilk and hindmilk samples from all four mothers.

Sequence	Start	Stop
IPVKQADSGSSEEKQLYNK	17	35
IPVKQADSGSSEEKQLYNKYPDAVATWLNPDPSQ	17	50
IPVKQADSGSSEEKQLYNKYPDAVATWLNPDPSQK	17	51
IPVKQADSGSSEEKQLYNKYPDAVATWLNPDPSQKQN	17	53
VKQADSGSSEEKQLYNKYPDAVATWLNPDPSQK	19	51
SKSKKFRRPDIQYPDATDEDITSH	169	192
SKSKKFRRPDIQYPDATDEDITSHMESEELNGAY	169	202
SKSKKFRRPDIQYPDATDEDITSHMESEELNGAYK	169	203
SKKFRRPDIQYPDATDEDITSHMESEELNGAYK	171	203
KFRRPDIQYPDATDEDITSHMESEELNGAYK	173	203
FRRPDIQYPDATDEDITSHMESEELNGAY	174	202
FRRPDIQYPDATDEDITSHMESEELNGAYK	174	203
RRPDIQYPDATDEDITSHMESEELNGAY	175	202
RRPDIQYPDATDEDITSHMESEELNGAYK	175	203
RPDIQYPDATDED	176	188
RPDIQYPDATDEDITSH	176	192
RPDIQYPDATDEDITSHMESEELNGAY	176	202
RPDIQYPDATDEDITSHMESEELNGAYK	176	203
PDIQYPDATDEDITSHMESEELNGAYK	177	203
DIQYPDATDEDITSH	178	192
DIQYPDATDEDITSHMESEELNGAYK	178	203
IQYPDATDEDITSHMESEELNGAYK	179	203
YPDATDEDITSH	181	192
ESEELNGAYK	194	203
AIPVAQDLNAPSDWDSRGKDSYETSQLDDQSAETHSHK	204	241
RKANDESNEHSDVIDSQELSK	248	268
HLKFRISHELDSASSEVN	297	314
FRISHELDSASSEVN	300	314
RISHELDSASSEVN	301	314

*“Start” and “stop” indicate the amino acid numbers for the beginning and end of the peptide within the protein sequence (counting the signal sequence)*.

**Table 4:** Peptides identified with a significantly higher abundance in hindmilk than foremilk.

Sequence	Protein	Start	Stop
LPIPQQVVPYPQRA	β-Casein	177	190
YPVTQPLAPVHNPISV	β-Casein	211	226
LAQPAVVLPVPQPEIMEVPKAKDT	β-Casein	84	107
STDRSPYEKVSAGNGGSSLSYTNPAVAATSANL	Mucin-1	1,223	1,255
RLQNPSESSEPIPLESREEY	α_S1_-Casein	26	45
LAQPAVVLPVPQPEIMEVPKA	β-Casein	84	104
DQQQGEDEHQDKIYPS	β-Casein	43	58
RQRNILREKQTDEIKDTR	α_S1_-Casein	51	68
LESREEYMNGMNR	α_S1_-Casein	39	51
RSPYEKVSAGNGGSSLSYTNPAVAATSANL	Mucin-1	1,226	1,255
IPLSPMGEDSAPR	Butyrophilin subfamily 1 member A1	495	507
AQPAVVLPVPQPEIMEVPKAKDTVYTK	β-Casein	85	111
EIPLSPMGEDS	Butyrophilin subfamily 1 member A1	494	504
SPYEKVSAGNGGSSL	Mucin-1	1,227	1,241
EEKAVADTRDQADGSRASVDSGSSEEQGGSSR	Polymeric immunoglobulin receptor	607	638
PMGEDSAPRDADTLH	Butyrophilin subfamily 1 member A1	499	513
SPYEKVSAGNGGSSLS	Mucin-1	1,227	1,242
PAVVLPVPQPEIMEVPK	β-Casein	87	103
NPTHQIYPVTQPLAPVHNP	β-Casein	205	223
LSSSEESITEYK	β-Casein	22	33
DSVDIFK	Bile salt-activated lipase	45	51
LPIIQKLEPQIA	Perilipin-2	66	77
YTKGRVMPVLK	β-Casein	109	119
TNPAVAATSANL	Mucin-1	1,244	1,255
PLSPMGEDSAPRD	Butyrophilin subfamily 1 member A1	496	508
AIPVAQDLNAPSDWDSRGKDSYETSQL	Osteopontin	204	230
NGFKSHALQLNNRQIR	Complement C4-A	1,337	1,352
DGREQEAEQMPEYRG	Butyrophilin subfamily 1 member A1	79	93
KEIPLSPMGEDSAPR	Butyrophilin subfamily 1 member A1	493	507
PVTQPLAPVHNPISV	β-Casein	212	226
IESLSSSEESITEYKQKVEK	β-Casein	19	38
LQNPSESSEPIPLESREEYMNGMN	α_S1_-Casein	27	50
QPLMQQVPQPIPQT	β-Casein	147	160
PAVAATSANL	Mucin-1	1,246	1,255
AIPVAQDLNAPS	Osteopontin	204	215
HQIYPVTQPLAPVHNPISV	β-Casein	208	226

*“Start” and “stop” indicate the amino acid numbers for the beginning and end of the peptide within the protein sequence (counting the signal sequence)*.

The peptides derived on average from 24.5 ± 0.8 proteins in the foremilk and 27.0 ± 0.8 proteins in the hindmilk (*P* = 0.127). In total, peptides from 42 proteins were identified. The peptides derived mostly from β-casein (51.1 ± 7.4% of total abundance), osteopontin (31.1 ± 11.3%), α_s1_-casein (11.1 ± 6.1%), polymeric immunoglobulin receptor (3.2 ± 1.4%), butyrophilin (2.6 ± 2.6%), mucin-1 (0.3 ± 0.3%), bile salt-activated lipase (0.1 ± 0.08%), fibrinogen α-chain (0.08 ± 0.07%), and perilipin-2 (0.1 ± 0.1%). The remaining proteins accounted for 0.3 ± 0.1% of total abundance. The highest number of peptides derived from β-casein, and more peptides were identified from β-casein in hindmilk (199 ± 9 peptides) than in foremilk (149 ± 9 peptides) (*P* = 0.0312), although there was no difference in abundance (Figure 2). The second highest number of milk peptides derived from osteopontin. The count of peptides from osteopontin was higher in hindmilk (121 ± 2) than foremilk (111 ± 2) (*P* = 0.0334), but there was no difference in abundance. α_s1_-Casein-derived peptides were higher in hindmilk than foremilk by count (65 ± 1 vs. 53 ± 1, *P* = 0.00184) and tended to be higher in hindmilk than foremilk by abundance (*P* = 0.0587). For mucin-1, both the count (*P* = 0.0138) and abundance (*P* = 0.0129) of peptides were higher in hindmilk than foremilk (19 ± 1 vs. 12 ± 1 for count). Peptides deriving from polymeric immunoglobulin receptor and butyrophilin did not differ in count or abundance between foremilk and hindmilk.

**Figure 2:** Count **(A)** and abundance **(B)** of peptides derived from either foremilk or hindmilk. Results are shown as least square means ± SE, *n* = 4. Asterisks (*) indicate significant differences between foremilk and hindmilk (*P* < 0.05). CASB, β-casein; OSTP, osteopontin; CASA1, α_s1_-casein; BT1A1, butyrophilin subfamily 1 member A1; PIGR, polymeric immunoglobulin receptor; CEL, bile salt-activated lipase; PLIN2, perilipin-2; MUC1, mucin-1; FIBA, fibrinogen α-chain; CASK, κ-casein; TRFL, lactoferrin.

The total number of peptides deriving from β-casein, osteopontin, and α_s1_-casein accounted for most of the peptide abundance—94.7 ± 1.2 and 91.9 ± 1.2% in foremilk and hindmilk, respectively. The peptides identified in foremilk and hindmilk were highly similar, shown for these three proteins from which most peptides were derived (Figures 3–5).

**Figure 3:** Count **(A)** and abundance **(B)** of peptides identified in breast milk mapped on the sequence of β-casein.

**Figure 4:** Count **(A)** and abundance **(B)** of peptides identified in breast milk mapped on the sequence of osteopontin.

**Figure 5:** Count **(A)** and abundance **(B)** of peptides identified in breast milk mapped on the sequence of α_s1_-casein.

### Protease Activity Prediction

To identify which of the known proteases in milk were involved in digestion of the foremilk and hindmilk, we used three bioinformatic approaches. Each peptide typically has two cleavage sites, unless the N-terminus or C-terminus of the peptide coincides with the N-terminus or C-terminus of the protein sequence. Foremilk and hindmilk had 879 ± 27 and 1,101 ± 27 cleavage sites, respectively.

At the P1 amino acid position, the amino acid most often present was lysine followed by arginine, alanine, and serine (Figures 6 and 7). All of these amino acids were present at more cleavage sites in hindmilk than foremilk by count. Compared to peptides with lysine, arginine, and alanine at P1, peptides with serine at P1 were much less abundant. Cleavage sites with a lysine and arginine at P1 correspond with the known site specificity for plasmin, KLK 6, KLK 11, and thrombin. Peptides with proline, valine, glutamine, asparagine, isoleucine, phenylalanine, and tryptophan at the P1 position were also significantly higher in hindmilk compared with foremilk, by count. Of these, tyrosine, asparagine, and isoleucine at the P1 position of cleavage sites correspond with the site specificity of elastase. By abundance, only serine (*P* = 0.0258) and leucine (*P* = 0.0004) at the P1 position were significantly greater in hindmilk compared to foremilk.

**Figure 6:** Count of peptides distributed according to their P1 and P1′ cleavage site of foremilk and hindmilk. Results are shown as least square mean ± SE, *n* = 4. Asterisks (*) indicate significant difference between foremilk and hindmilk (*P* < 0.05).

**Figure 7:** Abundance of peptides distributed according to their P1 and P1′ cleavage site of foremilk and hindmilk. Results are shown as least square mean ± SE, *n* = 4. Asterisks (*) indicate significant difference between foremilk and hindmilk (*P* < 0.05).

At the P1′ position of each cleavage site, the amino acids alanine (*P* = 0.0258), leucine (*P* = 0.0155), glutamic acid (*P* = 0.0473), proline (*P* = 0.0057), glutamine (*P* = 0.0115), tyrosine (*P* = 0–0249), aspartic acid (*P* = 0.0071), and methionine (*P* = 0.0253) were significantly higher in hindmilk than foremilk by count. Of these, only alanine at the P1′ position corresponds with one of our listed protease cleavage preferences (thrombin).

Though examining the P1 and P1′ amino acids can indicate matches with enzyme cleavage specificity, enzyme cleavage patterns are often more complex than their P1 and P1′ preferences. Two tools predict which proteases are most likely responsible for peptide cleavages based on a more complex cleavage specificity pattern. Based on data from EnzymePredictor analysis, plasmin was involved in the most cleavages by count in both foremilk and hindmilk (Table 5). There were no significant differences in the odds ratios (i.e., the likelihood of protease activity) for any of the proteases between foremilk and hindmilk. However, the C-terminal (*P* = 0.0007) and total cleavage counts (*P* = 0.0162) assigned to plasmin and the N-terminal (*P* = 0.0028) and total cleavage counts (*P* = 0.0085) assigned to elastase were higher in hindmilk compared with foremilk. Thrombin was only found to be responsible for one cleavage; however, the number of expected cleavages was low as well, resulting in a high odds ratio. KLK 6 and 11 are not available for search within Enzyme Predictor.

**Table 5:** Proteases involved in digestion of human milk proteins as predicted by enzyme predictor.

Enzyme		N-terminal cleavage count	C-terminal cleavage count	Total cleavage	Unique cleavage	No. of expected cleavages within the peptide	Number of proteins cleaved	Odds ratio
Plasmin	Foremilk	144.0 ± 4.6	194.0 ± 0.9	338.0 ± 5.1	0.0 ± 0.0	564.00 ± 13.63	19.50 ± 0.34	3.6 ± 0.1
	Hindmilk	161.0 ± 4.6	212.5 ± 0.9*	373.5 ± 5.1*	0.0 ± 0.0	682.50 ± 13.63*	19.75 ± 0.34	3.3 ± 0.1
Elastase	Foremilk	54.3 ± 1.6	52.5 ± 3.3	106.8 ± 2.7	0.0 ± 0.0	633.00 ± 18.63	11.50 ± 0.44	0.9 ± 0.0
	Hindmilk	74.8 ± 1.6*	55.3 ± 3.3	130.0 ± 2.7*	0.0 ± 0.0	801.00 ± 18.63*	14.25 ± 0.4*	0.9 ± 0.0
Thrombin	Foremilk	0.2 ± 0.2	0.0 ± 0.0	0.3 ± 0.2	0.3 ± 0.2	0.3 ± 0.2	0.3 ± 0.2	1.3 ± 2.9
	Hindmilk	0.5 ± 0.2	0.0 ± 0.0	0.5 ± 0.2	0.5 ± 0.2	0.5 ± 0.2	0.5 ± 0.2	8.1 ± 2.9

Results are shown as least square mean ± SE, *n* = 4. Asterisks (*) indicate significant difference between foremilk and hindmilk (*P* < 0.05).

Proteasix also predicted that plasmin cleaved the largest number of peptides in the dataset. By this analysis, there were no differences for any of the predicted protease activities between foremilk and hindmilk; however, cleavages assigned to elastase tended to be higher in hindmilk compared with foremilk (*P* = 0.0572) (Table 6). More cleavage sites were unassigned in hindmilk than foremilk (*P* = 0.0137), as only 15.5 ± 0.4% of potential cleavages were assigned by Proteasix in hindmilk compared with 17.6 ± 0.4% in foremilk. Several cleavage sites were assigned to two or more of plasmin, KLK 6 and thrombin as Proteasix was not able to distinguish among these enzymes for a number of the cleavage sites. On average, 14 cleavage sites overlapped between plasmin and thrombin, 3 overlapped between KLK 6 and plasmin, 1 overlapped between thrombin and KLK 6 and 1 cleavage site overlapped among all three enzymes.

**Table 6:** Proteases involved in digestion of breast milk proteins as predicted by Proteasix.

	Plasmin	Elastase	Thrombin	Kallikrein 6	Kallikrein 11	Unassigned
Foremilk	97.8 ± 1.2	25.0 ± 2.8	24.0 ± 1.4	7.5 ± 0.6	0.0 ± 0.0	718.3 ± 26.5
Hindmilk	100.3 ± 1.2	36.8 ± 2.8	24.08 ± 1.4	9.0 ± 0.6	0.0 ± 0.0	914.0 ± 26.5*

Results are shown as least square mean ± SE of the number of cleavages, *n* = 4. Asterisks (*) indicate significant difference between foremilk and hindmilk (*P* < 0.05).

A large portion of the identified peptides could not be assigned to a specific enzyme. However, several of these peptides matched other peptides with sequential removal of single amino acids. These could be potentially assigned to exopeptidase activity. N-terminal sequential removal of amino acids, potentially representing aminopeptidase activity, was significantly higher in hindmilk (357.0.5 ± 9.4) than foremilk (294.5 ± 9.4) (*P* = 0.0190) by count, but it was not higher by abundance (4.6 × 10^11^ ± 4.9 × 10^10^ vs. 3.7 × 10^11^ ± 4.9 × 10^10^). C-terminal sequential removal of amino acids, potentially representing carboxypeptidase activity, was similarly higher by count in hindmilk (384.0 ± 10.2 peptides) than foremilk (302.8 ± 10.2) (*P* = 0.0109), but not abundance (3.5 × 10^11^ ± 3.5 × 10^10^ vs. 2.7 × 10^11^ ± 3.5 × 10^10^).

### Bioactivity

Searching the MBPDB for identified peptide homology with known bioactive peptides revealed two peptides with 100% alignment to a known bioactive peptide (Table 7). These two peptides derived from β-casein f105-117 (SPTIPFFDPQIPK) and f185-211 (QELLLNPTHQIYPVTQPLAPVHNPISV), which were identified in 7 and 5 of the eight milk samples, respectively. β-Casein f105-117 can increase cell proliferation (29), and β-casein f185-211 is antimicrobial (30). The abundances of these two peptides were not different between the foremilk and hindmilk. With an 80% homology threshold, an additional five peptides matched to β-casein f105-117 and an additional 21 peptides matched to β-casein f185-211. The total abundance of the peptides with >80% homology to the antimicrobial β-casein f185-211 was higher in hindmilk than foremilk (*P* = 0.0429), but not the total count (*P* = 0.1602). Neither the total abundance nor the total count of the peptides with >80% homology to β-casein f105-117 differed between foremilk and hindmilk. This search also identified six peptides with >80% homology to known ACE-inhibitory peptides and one additional peptide with >80% homology to a known antimicrobial peptide.

**Table 7:** Bioactive peptides in human foremilk and hindmilk samples.

Query peptide	Protein	Bioactive peptide	Function	Alignment
QELLLNPTHQIYPVTQPLAPVHNPISV	β-Casein	QELLLNPTHQIYPVTQPLAPVHNPISV	Antimicrobial	100.0
NQELLLNPTHQIYPVTQPLAPVHNPISV	β-Casein	QELLLNPTHQIYPVTQPLAPVHNPISV	Antimicrobial	96.4
ELLLNPTHQIYPVTQPLAPVHNPISV	β-Casein	QELLLNPTHQIYPVTQPLAPVHNPISV	Antimicrobial	96.3
NQELLLNPTHQIYPVTQPLAPVHNPIS	β-Casein	QELLLNPTHQIYPVTQPLAPVHNPISV	Antimicrobial	96.3
QELLLNPTHQIYPVTQPLAPVHNPIS	β-Casein	QELLLNPTHQIYPVTQPLAPVHNPISV	Antimicrobial	96.3
LNQELLLNPTHQIYPVTQPLAPVHNPISV	β-Casein	QELLLNPTHQIYPVTQPLAPVHNPISV	Antimicrobial	93.1
LNQELLLNPTHQIYPVTQPLAPVHNPIS	β-Casein	QELLLNPTHQIYPVTQPLAPVHNPISV	Antimicrobial	92.9
ELLLNPTHQIYPVTQPLAPVHNPIS	β-Casein	QELLLNPTHQIYPVTQPLAPVHNPISV	Antimicrobial	92.6
NQELLLNPTHQIYPVTQPLAPVHNPI	β-Casein	QELLLNPTHQIYPVTQPLAPVHNPISV	Antimicrobial	92.6
LLNQELLLNPTHQIYPVTQPLAPVHNPISV	β-Casein	QELLLNPTHQIYPVTQPLAPVHNPISV	Antimicrobial	90.0
LLNQELLLNPTHQIYPVTQPLAPVHNPIS	β-Casein	QELLLNPTHQIYPVTQPLAPVHNPISV	Antimicrobial	89.7
LLNQELLLNPTHQIYPVTQPLAPVHNPI	β-Casein	QELLLNPTHQIYPVTQPLAPVHNPISV	Antimicrobial	89.3
LLLNPTHQIYPVTQPLAPVHNPIS	β-Casein	QELLLNPTHQIYPVTQPLAPVHNPISV	Antimicrobial	88.9
LLNPTHQIYPVTQPLAPVHNPISV	β-Casein	QELLLNPTHQIYPVTQPLAPVHNPISV	Antimicrobial	88.9
NQELLLNPTHQIYPVTQPLAPVHNP	β-Casein	QELLLNPTHQIYPVTQPLAPVHNPISV	Antimicrobial	88.9
LLNPTHQIYPVTQPLAPVHNPIS	β-Casein	QELLLNPTHQIYPVTQPLAPVHNPISV	Antimicrobial	85.2
LNPTHQIYPVTQPLAPVHNPISV	β-Casein	QELLLNPTHQIYPVTQPLAPVHNPISV	Antimicrobial	85.2
ALLLNQELLLNPTHQIYPVTQPLAPVHNPISV	β-Casein	QELLLNPTHQIYPVTQPLAPVHNPISV	Antimicrobial	84.4
LLNQELLLNPTHQIYPVTQPLAPVH	β-Casein	QELLLNPTHQIYPVTQPLAPVHNPISV	Antimicrobial	81.5
LNPTHQIYPVTQPLAPVHNPIS	β-Casein	QELLLNPTHQIYPVTQPLAPVHNPISV	Antimicrobial	81.5
NPTHQIYPVTQPLAPVHNPISV	β-Casein	QELLLNPTHQIYPVTQPLAPVHNPISV	Antimicrobial	81.5
NQELLLNPTHQIYPVTQPLAPVH	β-Casein	QELLLNPTHQIYPVTQPLAPVHNPISV	Antimicrobial	81.5
SPTIPFFDPQIPK	β-Casein	SPTIPFFDPQIPK	Stimulates cell proliferation	100.0
KSPTIPFFDPQIPK	β-Casein	SPTIPFFDPQIPK	Stimulates cell proliferation	92.9
SPTIPFFDPQIPKL	β-Casein	SPTIPFFDPQIPK	Stimulates cell proliferation	92.9
SPTIPFFDPQIP	β-Casein	SPTIPFFDPQIPK	Stimulates cell proliferation	92.3
LKSPTIPFFDPQIPK	β-Casein	SPTIPFFDPQIPK	Stimulates cell proliferation	86.7
SPTIPFFDPQIPKLTD	β-Casein	SPTIPFFDPQIPK	Stimulates cell proliferation	81.3
DTVYTKGRVMP	β-Casein	TVYTKGRVMP	ACE-inhibitory	90.9
KDTVYTKGRVMP	β-Casein	TVYTKGRVMP	ACE-inhibitory	83.3
TVYTKGRVMPVL	β-Casein	TVYTKGRVMP	ACE-inhibitory	83.3
PFFDPQIPK	β-Casein	PFFDPQIP	ACE-inhibitory	88.9
FFDPQIPK	β-Casein	PFFDPQIP	ACE-inhibitory	87.5
LRQAQEKFGKDKSPKFQL	Lactoferrin	WNLLRQAQEKFGKDKSPK	Antimicrobial	83.3
IYPSFQPQPLI	β-Casein	YPSFQPQPLIYP	ACE-inhibitory	83.3

Peptide abundance is shown as least square mean ± SE, *n* = 4. Asterisks (*) indicate significant difference between foremilk and hindmilk (*P* < 0.05). Indented peptide sequences are related to a peptide present with 100% homology to a known bioactive peptide.

Bioactivity prediction software (CAMPR3) predicted a higher number of antimicrobial peptides in hindmilk (81 ± 4) compared to foremilk (62 ± 4) (*P* = 0.0381). The abundance of these peptides tended to be higher in hindmilk than foremilk (*P* = 0.0927) (Table 7). However, the percentage of predicted antimicrobial peptides among the total identified peptides did not differ between foremilk (13.2 ± 0.6% by count, 1.9 ± 1.4% by abundance) and hindmilk (13.7 ± 0.6% by count, 4.3 ± 1.4% by abundance).

The count of general bioactive peptides as predicted by Peptide Ranker was also higher in hindmilk (65 ± 2) compared to foremilk (56 ± 2) (*P* = 0.0306). The abundance of these peptides tended to be higher in hindmilk than foremilk (*P* = 0.0773) (Table 7). However, the percentage of predicted bioactive peptides compared to the total did not differ between foremilk and hindmilk by count (11.7 ± 0.3 vs. 11.0 ± 0.3%, respectively). The percentage abundance of predicted general bioactive peptides compared to the total tended to be higher in hindmilk (13.4 ± 0.4%) than foremilk (11.8 ± 0.4%) (*P* = 0.0555).

## Discussion

The findings from this study show that hindmilk contained a higher total count of peptides than foremilk, with no difference in peptide abundance. The difference in count derived from higher counts of peptides from β-casein, osteopontin, α_s1_-casein, and mucin-1. The most abundant proteins in human milk are β-casein, α_s1_-casein, α-lactalbumin, lactoferrin, immunoglobulin A, lysozyme, and serum albumin (31). Though peptides derived from casein proteins were identified, no peptides were identified from α-lactalbumin, immunoglobulin A, lysozyme, or serum albumin and only a single peptide was identified from lactoferrin. These proteins thus may not be hydrolyzed inside the mammary gland, enabling their continued function in the neonatal gut. Overall, the peptides identified in foremilk and hindmilk were highly similar to each other. This protein-specific peptide release pattern is similar to results from past human milk peptidomic studies (7, 16, 17).

As milk was pumped directly into a mixture of antiproteases on ice, followed by immediate freezing to ensure that no proteolytic activity would occur in these milk samples post expression, peptides identified here represent the hydrolysis of proteins by proteases within the mammary gland. In the time between expressions, milk components gradually pool within the mammary gland. This time period provides the incubation time necessary for the initiation of protein hydrolysis. As the milk is held at body temperature and most of the enzymes are most active at body temperature, this environment provides ideal incubation conditions for these enzymes. The findings of the present study confirm findings of previous studies that peptides are present in mother’s milk due to intra-mammary proteolysis (15, 16).

As expression of milk takes 20–45 min, the additional exposure in the mammary gland in contact with proteases prior to expression of hindmilk compared with the foremilk could have allowed for additional proteolytic action—observed as higher counts of peptides in hindmilk. However, as the total peptide abundance did not differ, the effect of additional time in the mammary gland on peptide release is limited.

The higher counts of peptides in hindmilk compared with foremilk mostly came from peptides with a lysine, arginine, alanine, and serine at the P1 position. These amino acids also were overall those most often identified at the P1 position for each cleavage site. The amino acids arginine and lysine at P1 match the cleavage specificities for plasmin, KLK 6, KLK 11, and thrombin. These proteases have partially overlapping cleavage specificity, making it impossible to distinguish between them on the basis of P1 alone. However, EnzymePredictor and Proteasix, which both use more complex analyses of cleavage specificity, predict that plasmin was the most active protease in milk. Proteasix also found cleavages that matched to elastase, thrombin and KLK 6, suggesting that they are also involved in proteolysis within the mammary gland. However, no cleavage sites were assigned to KLK 11 within Proteasix. None of the predicted protease activities were significantly different between foremilk and hindmilk within Proteasix and EnzymePredictor.

Unassigned cleavage sites were higher in hindmilk than foremilk as shown by Proteasix, which could indicate that other proteases not examined in these prediction algorithms are active and responsible for the overall differences in peptide profile between foremilk and hindmilk. Cytosol aminopeptidase and carboxypeptidase B2 are exopeptidases known to be active in milk (12), and a previous study has confirmed there to be free amino acids in human milk (32), which may derive from the activity of these exopeptidases. These proteases could account for the high number of unassigned cleavages, as these enzymes are not available as options in EnzymePredictor and Proteasix. Indeed, in hindmilk a significantly higher number of identified peptides corresponded to sets of peptides with sequential removal of amino acids from the N- and C-termini compared with foremilk.

Hindmilk showed a higher abundance of peptides with > 80% homology to the known antimicrobial peptide β-casein f185-211 (QELLLNPTHQIYPVTQPLAPVHNPISV) than foremilk. This peptide was originally identified after *in vitro* digestion of human milk with the protease *Lactobacillus helveticus* PR4 (30). However, we have shown that this peptide is produced naturally in the mammary gland in the absence of external protease activity and thus immediately available in active form to the infant or for action within the mammary gland itself. In an agar well diffusion assay (33), β-casein f185-211 demonstrated inhibitory activity against the potentially pathogenic species *Escherichia coli, Enterococcus faecium, Bacillus megaterium, Listeria innocua, Salmonella* spp., *Yersinia enterocolitica*, and *Staphylococcus aureus*. Several of these bacteria are known to inhabit the gut and may lead to infections in the infant, especially for those in neonatal care settings (34, 35).

In addition, hindmilk showed a higher number of peptides predicted to be potentially bioactive and also tended to be higher in abundance. However, on a percentage basis compared with the total number of peptides identified in each sample, hindmilk and foremilk did not differ in the relative amounts of predicted bioactive peptides. A potential limitation of our study in comparing bioactive peptide abundance is the small sample size (*n* = 4). However, as most peptides were found to be the same across fore- and hindmilk, the findings are likely robust.

The nutrient content of breast milk is considered to be insufficient to meet the needs of early pre-term infants and is typically fortified with additional nutrients, including protein (36, 37). Despite this fortification, pre-term infants with very low birth weight commonly have postnatal growth failure, which is associated with numerous long-term health issues. To provide the most optimal nutrition, some neonatal intensive care units feed low birth weight pre-term infants mother’s hindmilk, as it is more energy dense, and preserve the foremilk by freezing for later use (21, 38, 39). Findings in the present study for milk of term mothers indicate that this practice may provide increased numbers of bioactive peptides to pre-term infants during hindmilk feeding should pre-term mothers’ fore- and hindmilks differ similarly. As bioactive peptides may help protect and guide the development of the neonate, this contribution could lead to improved outcomes. Therefore, the potential to alter infant nutrition due to differences in peptides between foremilk and hindmilk is possible; however, as there are few differences in overall peptide abundance, the overall effect regarding peptides is likely limited.

## Conclusion

The findings demonstrate that hindmilk contains a higher number of peptides than foremilk, including peptides with antimicrobial activity. However, peptide abundance both overall and from individual proteins was similar in foremilk and hindmilk.

## Ethics Statement

This study was carried out in accordance with and approval by the Institutional Review Board at Oregon State University. Informed consent was obtained from all mothers.

## Author Contributions

SN and DD planned the study. SN collected the samples. SN and RB conducted the experiments and data analysis. SN, RB, and DD prepared the manuscript. All authors read and approved the final manuscript.

## Conflict of Interest Statement

The authors declare that the research was conducted in the absence of any commercial or financial relationships that could be construed as a potential conflict of interest. The reviewer EF and handling editor declared their shared affiliation.

## Footnotes

^1^http://bioware.ucd.ie/~enzpred/Enzpred.php.

^2^http://proteasix.org/.
